# A Cross-Talk between TrkB and Ret Tyrosine Kinases Receptors Mediates Neuroblastoma Cells Differentiation

**DOI:** 10.1371/journal.pone.0001643

**Published:** 2008-02-20

**Authors:** Carla Lucia Esposito, Amelia D'Alessio, Vittorio de Franciscis, Laura Cerchia

**Affiliations:** 1 Istituto per l'Endocrinologia e l'Oncologia Sperimentale "G. Salvatore", Consiglio Nazionale delle Ricerche (CNR), Naples, Italy; 2 Cell Biology and Preclinical Models Unit, INT-Fondazione Pascale, Naples, Italy; 3 Dipartimento di Biologia e Patologia Cellulare e Molecolare “L. Califano”, Università di Napoli “Federico II”, Naples, Italy; University of Arkansas, United States of America

## Abstract

Understanding the interplay between intracellular signals initiated by multiple receptor tyrosine kinases (RTKs) to give the final cell phenotype is a major pharmacological challenge. Retinoic acid (RA)-treatment of neuroblastoma (NB) cells implicates activation of Ret and TrkB RTKs as critical step to induce cell differentiation. By studying the signaling interplay between TrkB and Ret as paradigmatic example, here we demonstrate the existence of a cross-talk mechanism between the two unrelated receptors that is needed to induce the cell differentiation. Indeed, we show that TrkB receptor promotes Ret phosphorylation by a mechanism that does not require GDNF. This reveals to be a key mechanism, since blocking either TrkB or Ret by small interfering RNA causes a failure in NB biochemical and morphological differentiation. Our results provide the first evidence that a functional transactivation between distinct tyrosine kinases receptors is required for an important physiological process.

## Introduction

Receptor tyrosine kinases (RTKs) are transmembrane proteins that in response to growth factors stimulate intracellular pathways that control most fundamental cellular processes including the cell cycle, cell migration, cell metabolism and survival, as well as cell differentiation and proliferation. All known RTKs become activated by the selective binding of dimeric ligands to their extracellular domains, resulting in their dimerization and autophosphorylation [1], [2]. However, there is accumulating evidence that enlarges the traditional view of growth factor receptors activation in that the receptor may be transactivated and, thus, tyrosine-phosphorylated by ligands which specifically bind to other membrane receptors. For example, it has been widely demonstrated the transactivation of the epidermal growth factor receptor (EGFR) by agonists for G protein-coupled receptors (GPCRs) and other extracellular stimuli unrelated to EGF-like ligands [3], [4]. Similar to EGFR, it has been shown that activation of Trk (tropomyosin-related kinase) receptor tyrosine kinases TrkA (P04629 Swiss-Prot accession number) and TrkB (Q16620 Swiss-Prot accession number) can also occur via a GPCR mechanism, without involvement of nerve growth factor (NGF, P01138 Swiss-Prot accession number) or brain-derived neurotrophic factor (BDNF, P23560 Swiss-Prot accession number) [5], [6], [7] thus indicating alternative modes of stimulating trophic functions in neuronal cells by linking different receptor signalling pathways.

As first example of intracellular cross-activation between RTKs, it has been shown that in cultures of sympathetic neurons the NGF receptor, TrkA, acts on Ret (rearranged during transfection, P07949 Swiss-Prot accession number) kinase by an intracellular mechanism that transactivates its catalytic domain whereas doesn't require ligand expression [8].

As demonstrated for brain tumor glioblastoma multiforme and other solid tumours, the co-activation of RTKs limits the efficacy of therapies targeting single receptors [9], thus a deeper insights in the inter-RTK signalling pathways is needed to find combination of therapeutic agents with increased anti-cancer efficacy.

Neuroblastoma is the most common solid tumor of childhood outside the central nervous system; it is made of neural crest cells that can occur at any point along the sympathetic ganglia or the adrenal medulla. Expression of neurotrophin receptors of Trk family is an important prognostic factor in NB and activation of different Trk receptors leads to variable clinical presentation and behaviour of the tumor [10], [11]. Differences in the expression pattern of the receptors or their downstream signalling components could in part explain the differences in favourable (in the case of TrkA) or unfavourable (in the case of TrkB) tumors. However, the cross-talk between the Trk receptors and other receptors on cell surface may influence the outcome of the NB cellular response. In NB cells it has been shown that the stably transfection of TrkB receptor results in enhancing neuroblastoma invasiveness via upregulating the expression of hepatocyte growth factor and its receptor TK, c-Met [12]. The need of cooperation between TrkA and Ret pathways has been shown in the HTLA230 neuroblastoma cells as critical to promote neuronal differentiation [13].

Furthermore, there is evidence in literature indicating that the Ret and TrkB signal pathways are associated with the process of NB differentiation [14]. Previous studies have shown that RA induces the neuronal differentiation of many human neuroblastoma cell lines. It has been reported that RA alone induces neurite extension in NB cells (SH-SY5Y, LAN-5 and KCNR cells) which have endogenous expression of BDNF, *via* induction of TrkB expression [15], [16]. The existence of an autocrine loop sustained by RA-treatment and involving increase of TrkB expression and its activation, has been demonstrated for KCNR cells [15]. Furthermore, in all these cell lines RA also induces Ret tyrosine kinase receptor expression [17] and we have recently demonstrated that in SK-N-BE cells, the RA-treatment induces a positive autocrine loop that sustains Ret activation and downstream signalling and depends on glial-derived neurotrophic factor (GDNF, P39905 Swiss-Prot accession number) expression and release. Ret stimulation in turn is crucial to mediate cell differentiation [18].

However, even if collectively these data indicate a central role of TrkB and Ret receptors in RA-induced cell differentiation, a clear understanding of their respective biological need is still lacking and the mechanism for their involvement in this process has been never clarified.

Here, we investigated the mechanism of Ret and TrkB involvement in differentiation of malignant NB cells. Our results demonstrate that the RA-induced differentiation of human NB cells depends on the signalling interplay by TrkB and Ret receptors. By promoting Ret phosphorylation in a GDNF-independent manner, the BDNF-stimulated TrkB, causes the induction of the neurite outgrowth and expression of differentiation-specific molecular markers. This is the first report that describes the need of a functional transactivation between two unrelated RTKs to cause the final cell phenotype.

## Results

### Effects of Ret expression and activation in RA-induced differentiation of human NB cell lines

In order to dissect the respective roles played by TrkB and Ret receptors in RA-dependent NB cells differentiation we first analysed the effects of disabling the function of Ret by small interfering RNA (siRNA) in SK-N-BE, LAN-5 and SH-SY5Y cells.

The treatment of the three cell lines with 10 µM RA for 3 days caused a dramatic increase in Ret protein and autophosphorylation levels that were reduced to basal upon transfecting with a siRNA targeting human Ret (Figure 1A, compare lanes 1 and 4 to lane 2, for the three cell lines), whereas a non-silencing control siRNA had no effect (compare lane 3 to 2). Interestingly, inhibiting Ret expression hampered the process of differentiation induced by RA as assessed by monitoring the levels of two proteins whose expression is up-regulated upon RA-induced differentiation in several NB cell lines, the nerve growth factor inducible protein (VGF) and the growth associated protein 43 (GAP-43) [18], [19], [20]. As shown in Figure 1B, silencing of Ret resulted in a drastic inhibition of the RA-dependent induction of VGF and GAP-43 (between 60% to 90–100% of inhibition for the three cell lines), as expected no effect was observed with the negative control siRNA. To further confirm that the Ret silencing was correlated with a significant impairment of the RA-induced NB cells differentiation, we determined the expression levels of tissue transglutaminase (tTG) an enzyme whose increase has been reported to mediate RA-induced cell differentiation in NB cells [18], [21], [22]. As shown (Figure 1B), even upon RA-treatment, in the Ret-interfered cells the levels of tTG were almost undetectable as in the absence of RA-treatment (compare lanes 4 to 1). In agreement with our previous findings in SK-N-BE [18] these results demonstrate that Ret is generally required to the RA-induced differentiation of human NB cells.

**Figure 1:** Ret activity is involved in RA-induced NB cell differentiation. (A) and (B) SK-N-BE (*left panels*), LAN-5 (*middle panels*) and SH-SY5Y (*right panels*) cells were either left untreated (lane 1) or RA-treated (lane 2); RA-treated cells were transfected with Ret specific siRNA (siRNARet in lane 4) or a non-silencing control siRNA (siRNAns in lane 3). C, mock-treated cells. (A) Cell lysates were immunoblotted with anti-pRet or anti-Ret antibodies. To confirm equal loading the filters were stripped and reprobed with anti-αtubulin? antibodies, as indicated. Quantitations are done on the sum of the two Ret-specific enhanced chemiluminescence bands of 170 and 150 kDa corresponding to different glycosylation states of Ret. Intensity of bands have been calculated using the NIH Image Program on at least two different expositions to assure the linearity of each acquisition. Fold values are expressed relative to the reference points, arbitrarily set to 1 (labelled with asterisk). (B) To follow biochemical cell differentiation lysates were immunoblotted with anti-VGF, anti-GAP-43 or anti-tTG antibodies. The filters were blotted with anti-αtubulin? antibodies to normalize the loaded proteins, as indicated. Quantitation and relative abundances are expressed relative to controls, arbitrarily set to 1 (see A). Blots shown in (A) and (B) are representative of at least four independent experiments.

### RA induces the expression of BDNF and its receptor TrkB that mediates NB cell differentiation

In apparent discrepancy with the results reported above, in human KCNR neuroblastoma cells an autocrine loop involving the activation of TrkB by its ligand BDNF mediates RA-induced differentiation [15].

Therefore, we determined whether TrkB receptor was involved in SH-SY5Y, LAN-5 and SK-N-BE cells responsiveness to RA. To this aim, we first evaluated the expression levels of TrkB and its primary ligand BDNF in the three cell lines. As shown in Figure 2A, the cells express the full-length TrkB and BDNF RNA following RA-treatment (*left panel*). Furthermore, SH-SY5Y, LAN-5 and SK-N-BE cells express low levels of TrkB protein and their ability to express high levels of the receptor is regulated by RA (*right panel*).

As previously reported for KCNR cells, we found that in SH-SY5Y and in LAN-5, the RA-treatment leads to an increase of TrkB phosphorylation, suggesting that the endogenous BDNF expressed by these cell lines is sufficient to stimulate the activity of its own receptor (Figure 2B, compare lane 2 to l, in *left* and *middle* panels). At difference, in SK-N-BE the increase in the level of the protein following RA-treatment was not accompanied by detectable stimulation of its activity (compare lane 2 to 1 in *right panel*). Furthermore, in agreement with previously report [15], the TrkB receptor in SH-SY5Y and LAN-5 cells is competent for exogenous BDNF stimulation (Figure 2C, compare lane 2 to 1 and lane 4 to 3, respectively). In contrast, in SK-N-BE, phosphorylation of TrkB was undetectable even in the presence of an acute stimulation with exogenous BDNF (Figure 2C, compare lane 6 to 5) thus indicating that in this cell line RA induces the expression of a non-functional TrkB receptor. It has been widely reported that, *in vivo*, TrkB is spliced to generate truncated receptors that lack the cytoplamic kinase domain and that are expressed at different degrees in NB cells and tumors [23]–[26].

**Figure 2:** RA-dependent induction of expression and activation of TrkB in NB cells. (A) *Left*, RNA isolated from RA-treated SH-SY5Y, LAN-5 and SK-N-BE cells was reverse transcribed and amplified as described in Materials and Methods. Samples loaded on the gel are as follows: lanes 1, 2 and 3 amplification of TrkB in SH-SY5Y, LAN-5 and SK-N-BE, respectively; lanes 4, 5 and 6 amplification of BDNF in SH-SY5Y, LAN-5 and SK-N-BE, respectively; lane 7 markers IX (Roche); lanes 8 to 13, RNA samples as in lanes 1 to 6 but in the absence of RT as negative controls. *Right*, Lysates from SH-SY5Y, LAN-5 and SK-N-BE, left untreated or RA-treated, were immunoblotted with anti-TrkB antibodies against the extracellular domain of the receptor. The molecular weights of full-length TrkB and hypothetical TrkB.T1 isoform are indicated. The membranes were stripped and re-probed with anti-αtubulin? antibodies to control equal loading. Blots shown are representative of at least five independent experiments. (B) SH-SY5Y (*left panels*), LAN-5 (*middle panels*) and SK-N-BE (*right panels*) cells were left untreated or treated with RA in the absence or in the presence of TrkB siRNA (siRNATrkB) or the negative control siRNAns, as indicated. Cell lysates were immunoprecipitated with anti-panTrk antibodies and analysed by Western blotting with anti-pTyr or anti-TrkB antibodies. Blots shown are representative of at least four independent experiments. (C) RA-treated SH-SY5Y, LAN-5 and SK-N-BE cells were left un-stimulated (lanes 1, 3 and 5) or stimulated with BDNF (lanes 2, 4 and 6). Cell extracts were immunoprecipitated with anti-panTrk antibodies and immonoblotted with anti-pTyr or anti-TrkB antibodies. Blots shown are representative of at least three independent experiments. In (A), (B) and (C), quantitation and relative abundances are expressed relative to controls, arbitrarily set to 1 (see legend to Figure 1A).

The truncated isoforms have been shown to act as dominant inhibitors on BDNF signalling by sequestering the full-length receptor in non-functional heterodimers [25]. It is plausible that a similar mechanism of competitive TrkB inhibition by a truncated isoform could occur in SK-N-BE cells. Whether the 95 kDa-molecular weight, clearly visible in the immunoblot with TrkB antibodies (Figure 2A, *right panel*), corresponds to the truncated TrkB.T1 isoform remains to be determined.

Next, we wondered whether the RA-mediated TrkB up-regulation and activation mediate cell differentiation. To this aim we treated the cells with a specific siRNA for TrkB that completely blocked the expression of TrkB protein in the three cell lines (Figure 2B, lanes 4). As shown in Figure 3A, blocking TrkB expression resulted in the suppression of RA-dependent biochemical differentiation in SH-SY5Y and LAN-5 cells (*left* and *middle panels*) as monitored by the levels of GAP-43, tTG and VGF. In agreement with the observation that SK-N-BE cells express a non-functional TrkB (see Figure 2B and C), silencing had no effect in this cell line (*right panel*). Furthermore, both in SH-SY5Y and LAN-5 the extent of inhibition of RA-dependent induction of these same differentiation markers was comparable to that observed by interfering with Ret (compare Figure 1B to Figure 3A).

**Figure 3:** TrkB mediates the RA-dependent differentiation in SH-SY5Y and LAN-5. SH-SY5Y (*left panels*), LAN-5 (*middle panels*) and SK-N-BE (*right panels*) cells were left untreated or treated with RA in the absence or in the presence of siRNATrkB or the negative control siRNAns, as indicated. (A) Cell lysates were immunoblotted with anti-GAP-43, anti-tTG or anti-VGF antibodies. Equal loading was confirmed by immunoblotting with anti-αtubulin antibodies. Quantitation and relative abundances are expressed relative to controls, arbitrarily set to 1 (see legend to Figure 1A). Blots shown are representative of at least four independent experiments. (B) to (K): Following RA-treatment, the percentage of neurite outgrowth was calculated and reported as histogram (K). Data are percentage of neurite bearing cells/total cells analyzed. Columns, average of three independent experiments. Microphotographs of cells are shown (B to J).

The same behaviour as referred to the biochemical differentiation was also observed by monitoring the neurite outgrowth following RA-treatment of the three cell lines (Figure 3B to K). Indeed, as expected, disabling the expression of TrkB completely blocked the RA-induced neurite outgrowth in SH-SY5Y (Figure 3D) and LAN-5 (Figure 3G) cells but had no effect on SK-N-BE cells morphology (Figure 3J).

Taken together, the results demonstrate that disabling the expression of either Ret or TrkB causes a failure in RA-dependent cell differentiation, thus raising the question of the existence of a cooperative cross-talk between TrkB and Ret in neuroblastoma cells.

### It does exist cooperation between TrkB and Ret to induce RA-dependent NB differentiation?

Based on the recent findings that demonstrate that TrkA is able to transactivate Ret [8], we asked whether active TrkB could as well induce the transactivation of Ret in NB cells.

To this aim, we decided to hamper the function of the TrkB receptor by siRNA and monitor the level of phosphorylation of Ret following RA-treatment of SH-SY5Y (Figure 4A, *left panel*) and LAN-5 cells (Figure 4A, *right panel*). As shown, transfecting both the cell lines with the TrkB-specific siRNA for 72 h inhibits RA-induced Ret activation, but not expression, at the same extent of treating the cells with Ret specific siRNA (compare lanes 4 to 5, *left and right panels*). As a negative control, a non-related siRNA was also transfected into the cells that had no visible effects on phosphorylation (lane 3, *left and right panels*). In contrast, TrkB phosphorylation was not affected by inhibition of Ret by siRNA (data not shown). Thus, these results are compatible with the existence of a transactivation mechanism triggered by TrkB activity and acting on Ret in a ligand-independent manner.

**Figure 4:** Existence of a cross-talk between TrkB and Ret in SH-SY5Y and LAN-5 cells. (A) RA-treated SH-SY5Y (*left panels*) and LAN-5 (*right panels*) cells were transfected with siRNATrkB (lane 4), siRNARet (lane 5) or negative control siRNAns (lane 3). C is referred to untreated cells (lane 1). Cell lysates were immunoblotted with anti-TrkB, anti-pRet, anti-Ret, or anti-GAP-43 antibodies, as indicated. The equal protein loading has been confirmed by immunoblotting with anti-atubulin? antibodies. (B) RA-treated LAN5, SH-SY5Y and SK-N-BE cells were left un-treated (lanes 2, 5 and 8, respectively) or treated with BDNF (lanes 3, 6 and 9, respectively). Lanes 1, 4 and 7 are mock-treated cells. Cell lysates were immunoblotted with anti-pRet or anti-Ret antibodies. To confirm equal loading the filters were stripped and reprobed with anti-αtubulin? antibodies. In (A) and (B), quantitation and relative abundances are expressed relative to controls, arbitrarily set to 1 (see legend to Figure 1A). Blots shown in (A) and (B) are representative of at least three independent experiments.

As predicted by these results, blocking TrkB activation and in turn Ret phosphorylation caused a failure in RA-dependent cell differentiation, monitored as inhibition of the RA-dependent induction of GAP-43 protein (Figure 4A, *left and right panels*).

These results strongly indicate that RA-induced overexpression and activation of TrkB in SH-SY5Y and LAN-5 cells is mediated by Ret activation and leads to neuroblastoma cells differentiation, indeed blocking TrkB expression prevents Ret activation and cell differentiation at the same extent reached by silencing the Ret receptor.

### Exogenous BDNF stimulation of LAN-5 and SH-SY5Y cells induces Ret activation

To further confirm that Ret activity in LAN-5 and SH-SY5Y cells is TrkB-dependent, we asked whether the Ret receptor could be transactivated by exogenous BDNF addition.

To increase TrkB and Ret expression, LAN-5 and SH-SY5Y were treated with RA for 72 h and cells were then stimulated with BDNF (50 ng/ml) for 10 min. As shown in Figure 4B, the BDNF acute stimulation of the cells led to an increase of Ret phosphorylation with respect to the un-stimulated cells of 2.75 and 4.8 folds for LAN-5 and SH-SY5Y cells, respectively (compare lane 3 to 2 and lane 6 to 5). As expected the BDNF stimulation of the cells does not modify the expression levels of Ret in RA-treated as well in mock treated cells. Consistently, the stimulation with BDNF of SK-N-BE does not affect the RA-induced phosphorylation of Ret (Figure 4B, compare lane 9 to 8) thus reflecting the absence of a functional TrkB expression in this cell line (see Figure 2C). This supports our above finding that the activation of Ret in RA-treated SH-SY5Y and LAN-5 cells is dependent on TrkB activity.

### The cross-talk mechanism stimulating Ret tyrosine kinase activity is GDNF-independent

We have previously demonstrated that in SK-N-BE cells (lacking of a functional TrkB receptor) RA-induced differentiation is preceded by the accumulation of Ret and GDNF, and that Ret activation depends on the synthesis and the extracellular secretion of GDNF [18]. For what it concerns LAN-5 and SH-SY5Y cells, our results indicate that Ret phosphorylation following RA-treatment is due exclusively or at least in large part to a GDNF-independent mechanism that requires TrkB activity. To further confirm these findings we blocked GDNF-dependent activation of Ret by two different inhibitors: 1) the D4 aptamer, that inhibits Ret activity by directly binding its extracellular domain [27], [18]; 2) a truncated Ret protein, the EC-Ret^wt^ peptide, that competes for binding to GDNF, thus depleting the culture medium of the functional ligand [28], [29], [18]. Indeed, if in LAN-5 and SH-SY5Y cells Ret is activated by a GDNF-independent mechanism, using these molecules should have not to affect RA-induced Ret phosphorylation and differentiation.

As shown in Figure 5, the treatment of SK-N-BE cells with D4 aptamer (Figure 5A, *left panel*, lane 3) or the soluble EC-Ret^wt ^protein (Figure 5B, *left panel*, lane 3) strongly inhibited Ret activation, while, in SH-SY5Y and in LAN-5 cells, any attempt to interfere with Ret stimulation either by using D4 (Figure 5A, *middle panel*, lane 3 and *right panel*, lane 3, respectively) or EC-Ret^wt^ (Figure 5B, *middle panel*, lane 3 and *right panel*, lane 3, respectively) failed and the levels of tyrosine phosphorylated Ret remained high. In addition, no inhibiting effect was observed by increasing neither the concentrations nor the incubation time of the aptamer or of the protein on the cells (not shown). As negative controls, we used a scrambled sequence of the D4 aptamer (D4Sc in the Figure 5A) and the recombinant EC-Ret protein lacking of the domains responsible of the functional interaction between Ret and the GFRα1/GDNF complex (EC-Ret^1-387^ in Figure 5B).

**Figure 5:** The RA-induced stimulation of Ret activity is GDNF-independent in SH-SY5Y and LAN-5 cells. (A) SK-N-BE (*left panels*), SH-SY5Y (*middle panels*) and LAN-5 (*right panels*) cells were left untreated (lane 1) or treated for the indicated incubation times with RA either in the absence (lane 2) or in the presence of D4 (lane 3) or D4sc (lane 4). Cell lysates were immunoblotted with anti-pRet, anti-Ret, anti-tTG or anti-VGF antibodies. Equal loading was confirmed by immunoblotting with anti-αtubulin antibodies. (B) SK-N-BE (*left panels*), SH-SY5Y (*middle panels*) and LAN-5 (*right panels*) cells were incubated either in the absence (lane 2) or in the presence of ECRet^wt^ (lane 3) or EC-Ret^1-387^ (lane 4) as indicated. Lanes 2 to 4, treatment with RA. Cell lysates were immunoblotted with anti-pRet or anti-Ret and and to confirm equal loading the filters were stripped and reprobed with anti-αtubulin? antibodies. In (A) and (B), quantitations were done as reported in legend to Figure 1A and relative abundances are expressed relative to controls, arbitrarily set to 1. Blots shown in (A) and (B) are representative of at least three independent experiments.

Further, in SH-SY5Y and LAN-5, the cell differentiation was unaffected by D4 treatment, thus mirroring the activation of Ret. Indeed, as shown in Figure 5A, in both SH-SY5Y and in LAN-5 cells, VGF and tTG levels were induced by RA and remained high in presence of D4 (compare lane 3 to 2 in *middle* and *right panels*, respectively). As expected, in SK-N-BE cells D4 inhibited VGF as well tTG RA-dependent increase (compare lane 3 to 2 in *left panel*, and 18).

On the basis of these results it is possible to conclude that in SH-SY5Y and LAN-5 cells, Ret is activated by a GDNF-independent mechanism. Furthermore, given that both the aptamer and the recombinant EC-Ret^wt^ interfere with Ret dimerization acting by the outside of the cell membrane, their inability to interfere with Ret suggests that in these cells, a cross-talk mechanism acting on Ret, stimulates its tyrosine kinase activity by an intracellular pathway.

## Discussion

Receptor tyrosine kinases stimulation is a tightly regulated process that involves high affinity binding by external ligand polypeptide growth factors. Even tough this is recognised as the main mechanism that regulates RTK activity, recent reports indicate that alternative ways of activation exist that implicate transactivation triggered by other unrelated membrane receptors in the cytoplasm.

Here we report for the first time that a physiological process, as the RA-induced differentiation, requires a novel transactivation mechanism which places Ret tyrosine kinase receptor downstream of TrkB receptor.

As previously reported [15], [17], [18] retinoic acid treatment of several human neuroblastoma cells is rapidly followed by a strong increase in the expression of both these transmembrane receptors that become activated in the absence of exogenously added BDNF and GDNF ligands. Here we show that at difference of SH-SY5Y and LAN-5 cells, upon RA-treatment, in SK-N-BE the TrkB protein even increased in expression levels is neither tyrosine phosphorylated nor competent for BDNF acute stimulation. On the other hand, Ret is induced and phosphorylated at comparable levels in the three cell lines.

Furthermore, we demonstrate that a functional TrkB receptor is needed for RA-mediated cell differentiation, indeed silencing TrkB causes a failure in morphological and biochemical cell differentiation in SH-SY5Y and LAN-5 whereas no effects were observed in SK-N-BE cells that express a non-functional TrkB receptor. On the other hand, we show that blocking Ret expression and activation by siRNA hampers as well the process of differentiation thus indicating that in LAN-5 and SH-SY5Y cells the concurrent activity of both receptors is needed for differentiation.

In this scenario, the fact that, in SK-N-BE, cell differentiation exclusively depends on Ret activation [18] raises the obvious question of by which mechanism TrkB and Ret cooperate in order to shift the NB cells toward a differentiated phenotype.

Given that silencing of Ret impairs NB differentiation in the three cell lines this indicates that Ret signalling is a common critical step for differentiation. For what it concerns LAN-5 and SH-SY5Y cells, our results establish that the RA-mediated Ret activation and cell differentiation are, in turn, dependent on TrkB activity, since inhibition of TrkB by siRNA significantly impairs Ret phosphorylation. Furthermore, we can exclude the presence of a GDNF-dependent mechanism of Ret activation since neither the D4 aptamer nor the EC-Ret^wt^ soluble protein reveal effective in inhibiting Ret phosphorylation following RA treatment of LAN-5 and SH-SY5Y cells. Indeed, the D4 aptamer interferes with the GDNF-mediated Ret dimerization and the EC-Ret^wt^ molecule competes for binding to GDNF thus depleting the culture medium of the functional ligand [27], [28], [29].

Taken together, our findings strongly indicate that at least two mechanisms can lead to stimulation of Ret activity by RA: the first, characteristic of SK-N-BE cells, lacking of a functional TrkB receptor, implicates the expression and secretion in the medium of GDNF thus providing maintenance of an autocrine loop that mediates cells differentiation (18 and current results); the second, in LAN-5 and SH-SY5Y cells, implicates that Ret activation is mediated by TrkB activity and occurs in the absence of GDNF stimulation. This indicates that a cross-talk mechanism between TrkB and Ret is functional in human NB cells. Furthermore, we show that the BDNF acute stimulation of SH-SY5Y and LAN-5 cells leads to Ret phosphorylation and transactivation in the absence of GDNF, thus confirming the existence of such inter-RTK signalling. In conclusion here we demonstrate that in the three NB cell lines, the RA-dependent Ret activation, both if GDNF-mediated (SK-N-BE) or TrkB-mediated (SH-SY5Y and LAN-5) is needed to induce cell differentiation since the outcome of blocking Ret phosphorylation is a failure in NB cell differentiation.

Two major mechanisms could explain the TrkB-dependent Ret activation. First, TrkB may heterodimerizes with Ret following BDNF stimulation. Second, TrkB, once phosphorylated by BDNF could in turn activate Ret by an intracellular way.

The heterodimerization of the platelet-derived growth factor receptor with EGFR [30], [31] or fibroblast growth factor receptor [32] and heterodimerization of insulin-like growth factor receptor and EGFR [33] are examples showing that cross-talk of different receptors may be mediated, at least in some cases, by their heterodimerization. This is unlikely to happen between TrkB and Ret on the basis of the following observations. The D4 aptamer inhibiting properties base on the capability of the RNA molecule to fold in a specific three-dimensional shape that binds at high affinity to Ret monomer and interferes with homodimerization and activation of the receptor [27]. Therefore, it is plausible that this molecule once bound to Ret monomer could obstacle as well Ret/TrkB dimerization. Our result showing that the D4 is unable to hamper RA-dependent Ret activation and differentiation of LAN-5 and SH-SY5Y cells, lends support to the second mechanism.

Furthermore, it has been demonstrated the existence of cross-talk between the signal pathways mediated by Ret and by another member of the Trk-family, the TrkA receptor, in developing sympathetic neurons, whereby increased Ret expression and phosphorylation takes place as a consequence of TrkA activation by NGF by intracellular mechanisms [8]. These can include down-regulation of protein tyrosine phosphatases or up-regulation of tyrosine kinases acting on Ret and/or up-regulation of adaptor protein that activates Ret in the absence of GDNF. Work is in progress to clearly understand the mechanism and molecules involved in Ret transactivation.

Here we demonstrate that the Ret receptor can be recruited by the TrkB receptor to function in the NB cells differentiation thus revealing a novel mechanism of functional cooperation between receptor tyrosine kinases. The understanding of the functional interplays between receptor is of major importance for the rationale design of new therapeutics in cancer.

## Materials and Methods

### Cell Culture and siRNA transfection

Human NB cell lines SK-N-BE (2), SH-SY5Y and LAN-5 (American Type Culture Collection, Manassas, VA) were grown in Dulbecco's modified Eagle medium supplemented with 2 mM L-glutamine, 10% heat-inactivated fetal bovine serum (Hyclone, Celbio, South Logan, UT), and 50 µg/ml gentamycin. All-*trans* RA (Sigma, St. Louis, MO) was dissolved (10 mM) in DMSO and diluted at 10 µM-final concentration in serum-containing culture medium. For BDNF acute stimulations, SH-SY5Y, LAN-5 and SK-N-BE (900.000 cells/10 cm-plate) were RA-treated for 72 h, serum starved for 4 h and then incubated for 10 min in the absence or in the presence of BDNF (Alomone Labs, Jerusalem, Israel) at a final concentration of 50 ng/ml.

Ret or TrkB gene silencing was established by transfection of high performance validated Ret siRNA [34] specifically targeting Ret exon-2 (5′-GGGAUGCUUACUGGGAGAAtt3′) or TrkB stealth siRNA (5′-AACUUAAGCAGAAACAGCAUUACCA) custom-designed by Invitrogen, into SK-N-BE(2), SH-SY5Y and LAN-5 NB cell lines. Cells (35.000 cells per 6 cm plate) were grown and overlaid with the transfection mixtures containing 100 nM Ret siRNA or 150 nM TrkB siRNA and Lipofectamine 2000 (Invitrogen, Carlsbad, CA) in Opti-MEM I reduced serum medium (Invitrogen). After 5-h incubation, complete culture medium containing 10 µM RA was added to the cells and incubation was prolonged up to 72 h. Controls were performed using a non-related siRNA that do not lead to the specific degradation of Ret and TrkB mRNA.

### Immunoprecipitation and western blot analysis

Cells were washed twice in ice-cold phospate-buffered saline (PBS), and lysed in buffer A (50 mM Tris-HCl pH 8.0 buffer containing 150 mM NaCl, 1% Nonidet P-40, 2 µg/ml aprotinin, 1 µg/ml pepstatin, 2 µg/ml leupeptin, 1 mM Na_3_VO_4_). Protein concentration was determined by the Bradford assay using bovine serum albumin as the standard. For immunoprecipitation analysis, cell extracts (500 µg) were incubated with anti-panTrk antibody (C-14) (Santa Cruz Biotechnology Inc, Santa Cruz CA) for 2 h at 4°C and then immunoprecipitated with protein A/G- agarose (Santa Cruz Biotechnology Inc, Santa Cruz CA) overnight at 4°C. Immunoprecipitates were washed three times with buffer A and denatured in Laemmli buffer for 5 min at 100°C. The cell lysates or immunoprecipitates were subjected to 8% SDS-PAGE. Gels were electroblotted into polyvinylidene difluoride membranes (Millipore Co., Bedford, MA), and filters were probed with the indicated primary antibodies: anti-Ret (H-300), anti-TrkB (H-181), anti-VGF (R-15) (Santa Cruz Biotechnology Inc, Santa Cruz CA); anti-(Tyr-phosphorylated) Ret (referred as pRet) (Cell Signaling, Beverly, MA); anti-phospho-tyrosine (referred as pTyr) (4G10, Upstate Biotechnology Incorporated, Charlottesville, VA); anti-GAP-43 (Zymed Laboratories Inc., South San Francisco, CA); anti-α-tubulin (DM 1A) (Sigma, St. Louis, MO); anti-tTG antibodies (kindly provided by G. Peluso CNR, Naples, Italy) [35]. Proteins were visualized with peroxidase-conjugated secondary antibodies using the enhanced chemiluminescence system (Amersham-Pharmacia Biosciences LTD, Uppsala, Sweden). Where indicated, filters have been stripped as described [28].

### Reverse Transcription-PCR analysis

10^6^ NB cells were plated on 10-cm dishes and treated with 10 µM RA for 72 h for analysis of full-length TrkB and BDNF mRNA. Amplification of glyceraldehyde-3-phosphate dehydrogenase (GAPDH) was used as control to normalize the levels of mRNA in all samples. Total RNA was isolated using a RNA extraction kit (Ambion Austin, TX). RNA (5 µg) was reverse transcribed for 60 min at 42°C in a 20 µl-volume reaction mixture containing 20 units of Moloney Murine Leukaemia Virus Reverse Transcriptase (M-MV-RT) (Roche, Basel, Switzerland) and random hexanucleotides (Amersham Pharmacia). The resulting cDNA fragments were used as PCR templates.

The following pairs of forward and reverse primer sets were used for amplification: TrkB, 5′-GAGCATCATGTACAGGAAAT-3′ and 5′-CTTGATGTTCTTCCTCATGT-3′ (PCR product size, 235 bp); BDNF, 5′-GCAACGGCAACAAACCACAACATTATC-3′ and 5′-GTCCCTGTATCAAAAGGCCAACTGAAG-3′ (PCR product size, 492 bp); GAPDH, 5′-CATCAAGAAGGTGAAGC-3′ and 5′-TCTTACTCCTTGGAGGCCAT-3′ (PCR product size, 240 bp).

Amplifications were performed by 30 cycles of PCR by using the following conditions: TrkB: 30 sec at 95°C; 30 sec at 57°C and 30 sec at 72°C; BDNF: 1 min at 94°C, 1 min at 60°C and 2 min at 72°C; GAPDH: 20 sec at 95°C, 30 sec at 58°C and 1 min at 72°C.

### Neurite Outgrowth Bioassay

NB cells were plated at equal density on 10-cm dishes. To evaluate the effects of TrkB gene silencing on morphologic cell differentiation, cells were transfected with TrkB-specific or non-related siRNA as reported in *Cell Culture and siRNA trasfection.* At 72 h of RA treatment, at least 15 random fields were photographed by a phase-contrast light microscope and 50 cells per frame were counted and scored as having neurites or not. A neurite was operationally defined as a process outgrowth that was long more than twice the diameter of cell body.

### Inhibitors of GDNF-dependent Ret activation

D4 is a 93-base 2′-fluoro-RNA-based aptamer that specifically bind the extracellular domain of Ret thus interfering with ligand-induced stimulation of its intrinsic tyrosine kinase activity [18]. A scrambled sequence of D4 (D4sc) is used as control.

The entire Ret receptor extracellular portion (EC-Ret^wt^) and the protein containing just the first three NH_2_-terminal cadherin-like domains of EC-Ret^wt^ (named EC-Ret^1-387^) were produced as reported previously [28], [29].

To assess the effects of RNA aptamers and of EC-Ret proteins on Ret activity, SK-N-BE, SH-SY5Y and LAN-5 cells (160.000 cells/3.5 cm-plate) were treated for 18 h with 1 ml-culture medium containing 10 µM RA plus 50 µg of indicated EC-Ret or 1600 nM of indicated aptamers after a short denaturation-renaturation step. To evaluate the effects of D4 aptamer on cell differentiation, cells were incubated in 12-well cell plate with 10 µM RA together with 3 µM aptamer for 72 h. The used RNA concentrations ensure the continuous presence of a concentration of at least 200 nM, which takes into account the 6 h-half life of the D4 aptamer in 10% serum. This concentration is effective in inhibiting Ret activity as previously reported [18], [27].
